The article "Modeling and Analysis of the Influence of Cultural Differences on English Learning from the Perspective of the Cultural Community" was published in 2022. Journal: J Environ Public Health.

# Modeling and Analysis of the Influence of Cultural Differences on English Learning from the Perspective of the Cultural Community

**DOI:** 10.1155/2022/4674721

**Published:** 2022-09-26

**Authors:** Bin Tang, Haonan Zhang, Yuqin Jiang

**Affiliations:** School of Foreign Languages, Research Center for Applied Transportation and Engineering, East China Jiaotong University, Nanchang, Jiangxi, China 330013

## Abstract

A model of the influence of cultural differences on English learning from the perspective of the linguistic and cultural community based on data feature decomposition and fusion clustering is proposed. The new knowledge and the old knowledge are connected through the optimal control of the learning model. By decomposing relevant data through data features and fusion clustering algorithm, the impact of cultural differences on English learning can be modeled and analyzed from the perspective of language and cultural community. The simulation results show that the data fusion performance of the impact model of this method on English learning is good, and the quantitative analysis results are accurate and reliable. According to the results of visual data, targeted interventions were carried out for teachers, learners, and teaching managers.

## 1. Introduction

Teachers have always played an important role in the process of English teaching and in the establishment of English language and cultural status. In this process, higher requirements are put forward for teachers' teaching skills and academic abilities, so teachers need to constantly improve their teaching quality [1–3]. In college English teaching, the spread of English language and culture has always been in a one-way state, with teachers transmitting relevant knowledge to students, while two-way interactive communication has always been absent. If this situation wants to be changed, first, the current situation of college English language and culture learning should be understood, and both teachers and students should pay attention to the importance of establishing the status of English language and culture. Teachers and students need to increase interactive teaching links, so that students can better understand English language and culture through practice, and teachers also need to improve the teaching content and process, so as to speed up the establishment of English language [4–6]. Studying the influence of cultural differences on English learning from the perspective of language and cultural community is of great significance to improving English learning and education quality.

Among the traditional methods, there are mainly parametric methods based on ambiguity detection and feature vector fusion and the influence of cultural differences on English learning from the community perspective [7, 8]. Reference [9] proposes a model to guide English learning interest based on multivariate quantitative recursive analysis. By using descriptive statistical analysis, the constraint parameters of guiding English learning interest are constructed. And the guiding model of English learning interest in microclasses is transformed into a multiple linear regression model. Construct each explanatory variable for robust regression analysis. The model analyzes the correlation between the guidance of English learning interest and the learning quality, and evaluates the students' English learning interest and predicts the quality of English learning by means of multivariate quantitative recursive analysis. In this method, the guiding role of English learning interest in the microclassroom model is simulated. The results of quantitative analysis are accurate, the evaluation of English learning interest is reliable, and the effect of improving English learning quality is obvious. However, this method is computationally expensive. Reference [10] uses multilevel modeling to investigate the development of oral English complexity of Chinese learners in one academic year. And learners' individual development trajectory and group development trend are simulated. It is found that the development process of individual learners' oral complexity in different dimensions is different. At the group level, the unit length of learners increased significantly; the master — slave relationship increased weakly, and the length of phrases decreased slightly. The study further uses change point analysis and semistructured interviews to explore the development trend and reasons of learners' complexity in high-growth group and low-growth group. The results show that under the influence of different learning motivation and emotion, the complexity development of the high-growth group shows an upward trend after the change point and that of the low-growth group shows a downward trend. This method shows that the multilevel modeling method can deepen the understanding of the oral development process and the research results are helpful for teachers to better design oral teaching tasks.

The article "Modeling and Analysis of the Influence of Cultural Differences on English Learning from the Perspective of the Cultural Community" was published in 2022. Journal: J Environ Public Health.

In view of the above problems, this paper proposes a model of the impact of cultural differences on English learning from the perspective of language and culture community, based on data feature decomposition and fusion clustering. Using the differential semantic feature detection method, the index parameter distribution model of the impact of cultural differences on English learning from the perspective of language and cultural community is constructed. The relevant data collected on the English learning platform, including learners' learning logs and learning achievements, are used to realize the modeling and quantitative analysis of the impact of cultural differences on English learning from the perspective of language and cultural community. The experimental results show that this method is superior in improving the modeling ability of the influence of cultural differences on English learning.

## 2. Clustering Algorithm Theory

Any clustering algorithm has certain assumptions about the data set itself. If the distribution of the data set itself does not conform to the preassumption, the result of the algorithm will be meaningless, even it can be said that the result just gives a wrong distribution or imposes a fictitious distribution on the data set. Clustering combines the results obtained by different algorithms or using different parameters in the same algorithm, so as to obtain better results than a single algorithm.

In clustering fusion, multiple cluster members of the data set are generated first, and then, the clustering results of these cluster members are merged by consensus function. We select different initial points randomly and run the *k*-means algorithm several times, so as to generate the required cluster members. We use random sampling method to generate data subsets and then use *k*-means algorithm to generate clusters for each data subset, so as to get cluster members. Random projection is used to project high-dimensional data into low-dimensional space, and several data subsets are obtained by multiple projections. Then, the EM clustering algorithm is used to cluster each projection subset, so as to obtain cluster members. By selecting different algorithms, selecting different initial values for an algorithm, selecting different subsets of objects, selecting different subsets of features, and projecting them into the data subspace, cluster members are generated. The algorithm is used to measure the similarity between data points. Points larger than 0.5 in the matrix are considered to belong to the same class in the final clustering results.

The clustering fusion algorithm has excellent average performance in various fields and experiments and can adapt to most fields and experiments. Moreover, the noise data and abnormal data have little impact on the results of clustering fusion. Therefore, the clustering algorithm has the advantages of robustness, adaptability, and stability. Therefore, the learning model constructed by clustering fusion algorithm is applied in this paper, which provides a basis for subsequent relevant data analysis.

The article "Modeling and Analysis of the Influence of Cultural Differences on English Learning from the Perspective of the Cultural Community" was published in 2022. Journal: J Environ Public Health.

## 3. Influence of Cultural Differences on Parameter Distribution and Information Preprocessing

### 3.1. Influence Parameter Distribution and Information Preprocessing

The data of the process model of the influence of cultural differences on English learning mainly come from the following: (1) Learners make records through platforms, mobile terminals, software, etc. These data can reflect the interaction process between learners and platforms and can be used to analyze learners' learning behavior. (2) Curriculum, learning data, and data related to learners' learning. Managers can analyze these two kinds of data to provide feedback for teachers' teaching and students' learning.

These two kinds of data are analyzed by means of conceptual cognition, social network analysis, influence, and success or failure signals, followed by data tracking and prediction to form technical, social, and teaching individualization or adaptation. Learning analysis and process model are used to provide theoretical basis for junior high school English personalized learning instructional design supported by network teaching platform [11].

A feature matching model of the index parameters of the influence of cultural differences on English learning from the perspective of linguistic and cultural communities is constructed by combining semantic feature analysis and fusion scheduling method, which makes it the rough set feature quantity of the index parameters of the influence of cultural differences on English learning from the perspective of linguistic and cultural communities [12–14]. The specific construction process is sh`own in Figure 1.

According to the information fusion matching results of feature layers, a deep hash coding algorithm is adopted [15, 16]. In this paper, the depth feature detection is carried out on the index parameters of the influence of cultural differences on English learning from the perspective of linguistic and cultural communities. Moreover, the gradient values of the index parameters of the influence of cultural differences on English learning from the perspective of each linguistic and cultural communities are calculated. Using the inherent sparseness of data, the convergence value of depth hash coding is obtained as follows:

(1) $$\begin{array}{c} P\left(\underset{T⟶\infty }{\lim}\bar{x_{T}}=K\right)=1, \end{array}$$

wherein $\bar{x_{T}}$ represents the correlation parameter between cultural differences and English learning correlation feature set from the perspective of linguistic and cultural communities. *k* is the scale of random features. Additionally, *Q*(*x*_*i*_, *y*_*i*_) is the frame sequence moment of the index parameters of cultural differences' influence on English learning from the perspective of linguistic and cultural communities. According to the parameter fusion results of the index parameters of cultural differences' influence on English learning from the perspective of linguistic and cultural communities [17–19], the joint feature distribution set of the index parameters of cultural differences' influence on English learning from the perspective of linguistic and cultural communities is expressed as follows:

(2) $$\begin{array}{c} F\left(t\right)=X_{p}\left(u-v\sin a\right)=\frac{3}{{\left(N+1\right)}^{2}}x\left(N+1\right)x^{3}\left(N+1-\tau \right), \end{array}$$

wherein *X*_*p*_ is the source information of semantic distribution of index parameters of cultural differences on English learning from the perspective of linguistic and cultural communities. *u* is the joint distribution feature quantity of index parameters of cultural differences on English learning from the perspective of linguistic and cultural communities. Moreover, *v* is the basis function of sparse representation classification model. We suppose *i* = 1. Read in the related features of cultural differences and English learning from the perspective of linguistic and cultural communities in the first frame and combine the coding of related features of cultural differences and English learning from the perspective of linguistic and cultural communities to obtain the output fuzzy feature code element sequence as follows:

(3) $$\begin{array}{c} \left\{\begin{array}{c} p_{th}^{\left(b_{\text{in}t}\right)}=C_{t}\underset{x_{i}\in w}{\sum }k\left(\left\|x_{i}\right\|\right)\delta \left(h\left(x_{i}\right)-b_{\text{in}t}\right),\\ p_{te}^{\left(b_{ine}\right)}=C_{e}\underset{x_{i}\in w}{\sum }k\left({\left\|x_{i}\right\|}^{2}\right){his}_{x_{i}}\delta \left(v_{x_{i}}-b_{ine}\right), \end{array}\right. \end{array}$$

wherein *C*_*t*_ = *C*_*e*_ = (1/∑_*x*_*i*_∈*w*_*k*(‖*x*_*i*_‖^2^)) represents the depth information parameter of the influence of cultural differences on English learning from the perspective of linguistic and cultural communities. *b*_in*e*_ ∈ [1, *M*] is the attribute category of linguistic and cultural communities. *h*(*x*_*i*_) is the greedy function of mixed structure. *b*_in*t*_ is the symbol transmission speed of characteristic frames from the perspective of linguistic and cultural communities. *b*_*ine*_ is the frame conversion rate. ‖*x*_*i*_‖ is the distance between clusters of sparse features, which represents a European distance.

The article "Modeling and Analysis of the Influence of Cultural Differences on English Learning from the Perspective of the Cultural Community" was published in 2022. Journal: J Environ Public Health.

The feature distribution quantity *u* in the joint feature distribution set obtained by formula (2) can determine the distribution of parameters. The larger the *u* is, the more obvious the distribution of joint features is. Therefore, the influence of cultural differences on the distribution of English learning parameters can be judged.

The new and old knowledge will be connected to form new knowledge experience, and the relevant data collected on the English learning platform. Learners' learning logs and learners' learning achievements will be analyzed in summary, so as to realize the integration of the indicators and parameters of the influence of cultural differences on English learning from the perspective of linguistic and cultural communities.

### 3.2. Information Characteristic Analysis of Influencing Index Parameters

The collected characteristic information of the influence of cultural differences on English learning from the perspective of linguistic and cultural communities is restructured, the feature distribution set is extracted, and the influence of cultural differences on English learning from the perspective of linguistic and cultural communities is realized by using the support vector machine algorithm. The specific process is shown in Figure 2.

According to the depth feature weighting training [20–22], the weighted aggregate output function of the influence of cultural differences on English learning from the perspective of linguistic and cultural communities is obtained as follows:

(4) $$\begin{array}{c} E_{Snake}=\overset{N-1}{\underset{0}{\sum }}\left[E_{\mathrm{int}}\left(vi\right)+E_{\mathrm{ext}}\left(vi\right)\right] \end{array}$$

wherein *V*_*i*_ is the morphological function of weighted aggregation of indicators and parameters of cultural differences' influence on English learning from the perspective of linguistic and cultural communities. *i* = 0, 1, ⋯*N* − 1 is the collection of characteristic points of cultural differences' influence on English learning, and *E*_ext_(*vi*) is the sparse scattered point set of cultural differences' influence on English learning. The aggregated output of sparse expression characteristic distribution of cultural differences' influence on English learning is *G* [23, 24], as shown below:

(5) $$\begin{array}{c} G_{t}={AF}_{t-1}+t, \end{array}$$

wherein *F*_*t*_ = [*x*_*t*_, *y*_*t*_]^*T*^ is the correlation characteristic value of the T-frame of the teaching resources of the correlation between cultural differences and English learning from the perspective of linguistic and cultural communities and *A* is the output amplitude. The semantic correlation distribution model of the index parameters of the influence of cultural differences on English learning from the perspective of linguistic and cultural communities is constructed. In addition, the distribution of output search trajectories is obtained, as shown below:

(6) $$\begin{array}{c} \text{trace}\left(x,y,\sigma^{\left(n\right)}\right)>\text{trace}\left(x,y,\sigma^{\left(1\right)}\right)\;l\in \left\{n-1,n+1\right\}, \end{array}$$

wherein trace(.) represents the fusion parameter of the index parameters of the influence of cultural differences on English learning from the perspective of linguistic and cultural community. Furthermore, the iterative function of the index parameters of the influence of cultural differences on English learning from the perspective of linguistic and cultural communities is obtained as follows:

(7) $$\begin{array}{c} X_{t}={AX}_{t-1}+t, \end{array}$$

wherein *X* = [*x*_*t*_, *y*_*t*_]^*T*^ is the frame distribution set of training characteristics from the perspective of linguistic and cultural community. The output clustering matrix of the index parameters of the influence of cultural differences on English learning from the perspective of linguistic and cultural communities is obtained as follows [25–27]:

(8) $$\begin{array}{c} H=\left[\begin{array}{cc} L_{xx}\left(x,\sigma \right) & L_{xy}\left(x,\sigma \right)\\ L_{xy}\left(x,\sigma \right) & L_{yy}\left(x,\sigma \right) \end{array}\right], \end{array}$$

wherein  *Lxx*(*x*, *σ*) is the characteristic matching coefficient of the index parameters of the influence of cultural differences on English learning from the perspective of linguistic and cultural communities. Moreover, *Lxy* and *Lyy* are the characteristic components of the index parameters of the influence of cultural differences on English learning from the perspective of linguistic and cultural communities in different aggregation directions.

The article "Modeling and Analysis of the Influence of Cultural Differences on English Learning from the Perspective of the Cultural Community" was published in 2022. Journal: J Environ Public Health.

## 4. Modeling and Optimizing

### 4.1. Data Feature Decomposition and Fusion Clustering Algorithm

The index parameter distribution model of the influence of cultural differences on English learning from the perspective of linguistic and cultural communities is constructed by using the differential semantic feature detection method. Under constructivism, the deep learning model of the influence of cultural differences on English learning, from the perspective of linguistic and cultural communities, is established by using the methods of knowledge ontology structure reconstruction and semantic feature fusion cluster analysis. And the collected correlation between cultural differences and English learning from the perspective of linguistic and cultural community is decomposed by sparsity features. The specific process is shown in Figure 3.

According to the hash coding results of the index parameters of cultural differences on English learning from the perspective of linguistic and cultural community, information reorganization is realized. In addition, the coding model of support vector machine is constructed according to the information reorganization structure. By using cluster analysis method, it is found that the cluster centers of the index parameters of cultural differences on English learning from the perspective of linguistic and cultural communities are *M*_*i*_ and *M*_*j*_, and the structural sparseness of data is represented by complexity. The reliability matching degree of cultural differences on English learning index parameters from the perspective of linguistic and cultural communities is Clustdist(*M*_*i*_, *M*_*j*_), and the corner information of cultural differences on English learning index parameters from the perspective of linguistic and cultural communities is extracted. The hierarchical alignment mechanism from coarse to fine is expressed as follows:

(9) $$\begin{array}{c} R_{1}\left(k\right)=R_{2}\left(k\right)\exp\left(-j\omega_{0}T_{p}/2\right),\;k=0,1,\cdots ,\left(N-3\right)/2, \end{array}$$

(10) $$\begin{array}{c} R_{2}\left(k\right)=A_{k}\exp\left(j\varphi_{k}\right),\;k=0,1,\cdots ,\left(N-3\right)/2, \end{array}$$

wherein *R*_2_(*k*) is the correlation characteristic component between cultural differences and English learning from the perspective of linguistic and cultural community. *T*_*p*_ is the collection time interval of Gaussian mixture sparse characteristic distribution. *ω*_0_*T* is the joint component, *A*_*k*_ is the kernel matrix of Mahalanobis distance. *ω*_0_ is the distance measurement parameter, and *N* is the weighting coefficient. Based on the semantic information detection results of the index parameters of the influence of cultural differences on English learning from the perspective of linguistic and cultural communities and the analysis results of the moment invariants of the correlation between cultural differences and English learning from the perspective of multiview attribute coding linguistic and cultural communities, the generalization model parameters of the vector machine regression model are as follows:

(11) $$\begin{array}{c} \varphi \left(X_{k},t_{i}\right)=G\left(\left\|X_{k},t_{i}\right\|\right)=\exp\left(-\frac{1}{2{\sigma_{i}}^{2}}{\left\|X_{k},t_{i}\right\|}^{2}\right)=\exp\left(-\frac{1}{2{\sigma_{i}}^{2}}\overset{M}{\underset{m-1}{\sum }}{\left(x_{km}-t_{im}\right)}^{2}\right) \end{array}$$

wherein *t*_*i*_ = [*t*_*i*1_, *t*_*i*2_, ⋯, *t*_*iM*_] is the discrete sequence of the index parameters of the influence of cultural differences on English learning from the perspective of linguistic and cultural community and *σ*_*i*_ is the iterative function of maximum likelihood estimation. The new curriculum standard requires a diversified evaluation system to promote students' all-round development. Different students have different interests and different learning styles. In teaching evaluation, students should not only be evaluated by a single examination method. Through the investigation of students' personalized contact opportunities and understanding methods, personalized learning in teaching is expected to be better understood.

The article "Modeling and Analysis of the Influence of Cultural Differences on English Learning from the Perspective of the Cultural Community" was published in 2022. Journal: J Environ Public Health.

### 4.2. Model Optimization Design

In the modeling of influence relationship, by controlling the distribution resources of cultural differences, the resources are selected and developed in the form of combining original resources with generative resources. We include answering materials, teachers' answers to common problems, students' discussion and sharing of personality problems, teachers' evaluation and summary of personality problems, and evaluation forms. Q&A material is a summary of the problems that teachers have with students after they preview. For the common problems of class students, teachers will focus on answering them in class. For the individual problems, teachers will discuss them in groups, and then, teachers will evaluate and summarize the results of students' discussions. Students will evaluate themselves and their classmates according to the contents in the evaluation form, extracting the frame recombination sequence of the correlation features between cultural differences and English learning from the perspective of linguistic and cultural community, and obtaining the robust multimodal multivariate sparse features, which are expressed as follows:

(12) $$\begin{array}{c} r_{1}\left(n\right)=r_{2}\left(n\right)\exp\left(-j\omega_{0}T_{p}/2\right),\;n=0,1,\cdots ,\left(N-3\right)/2, \end{array}$$

(13) $$\begin{array}{c} r_{2}\left(n\right)=A\exp\left[j\left(\omega_{0}nT+\theta \right)\right],\;n=0,1,\cdots ,\left(N-3\right)/2, \end{array}$$

wherein *N* is the sampling length of the correlation features between cultural differences and English learning from the perspective of linguistic and cultural community, *ω*_0_ is the symbol distribution interval of the evaluation feature sequence of students' discussion and sharing of personality problems and teachers' discussion of personality problems, and *T* is the maximum sampling length.

By analyzing the column vectors in the dictionary, this paper constructs an average segmentation model of the index parameters of the influence of cultural differences on English learning from the perspective of linguistic and cultural communities, which is expressed as follows:

(14) $$\begin{array}{c} \bar{x_{T}}=\frac{1}{T}\overset{T}{\underset{i=1}{\sum }}x_{i}, \end{array}$$

wherein *x*_1_, *x*_2_, *x*_3_ ⋯ *x*_*T*_ is the feedback sequence of formative evaluation from the perspective of linguistic and cultural community and *_T_* is the time delay parameter of linguistic and cultural community perspectives in series.

The article "Modeling and Analysis of the Influence of Cultural Differences on English Learning from the Perspective of the Cultural Community" was published in 2022. Journal: J Environ Public Health.

We construct a recombination model of the index parameters of the influence of cultural differences on English learning from the perspective of linguistic and cultural communities and obtain the joint measurement component of *N*_*l*_, and the calculation formula is shown as follows:

(15) $$\begin{array}{c} N_{l}=\left\{\begin{array}{cc} 1 & l=0,L,\\ \left[2\pi \cdot \frac{D}{2}\cdot \sin\eta /l_{triangle}\right] & 1, \end{array}\right. \end{array}$$

wherein *l*_*triangle*_ = *π* · *D*/2*L* represents the Retinex corner parameter value of the index parameter of the influence of cultural differences on English learning from the perspective of linguistic and cultural community. Moreover, *k* = 1, 2, ..⋯, *n*, *zk* ∈ *w*^*s*^, *ak* ∈ {1, 2, ⋯, *R*} is the Gaussian mixture sparse feature quantity. We establish a feature channel for quick retrieval of the index parameter information of the influence of cultural differences on English learning from the perspective of linguistic and cultural communities. According to the distributed fusion of edge features and frame sequence reorganization of the index parameter information of the influence of cultural differences on English learning from the perspective of linguistic and cultural communities, the comprehensive feature parameter is as follows: the test output result of the index parameter of the influence of cultural differences on English learning from the perspective of multilingual cultural community is shown as follows:

(16) $$\begin{array}{c} \overset{.}{\sigma_{i}}=\left\{\begin{array}{c} \mu \sin\frac{\pi e}{2\mu },\left|e_{i}\right|<\mu \\ \mu ,\left|e_{i}\right|\geq \mu -\mu ,\left|e_{i}\right|\leq -\mu \end{array}\right., \end{array}$$

wherein *σ*_*x*_, *σ*_*θ*_ and *e*_*i*_ represent the fitness parameter of the index parameter fusion of cultural differences on English learning from the perspective of linguistic and cultural community and represent the minimum augmented Lagrange function. Thus, we realize the fusion of the index parameters of cultural differences on English learning from the perspective of linguistic and cultural communities. Relevant data collected on the English learning platform, including learners' learning logs and learning achievements, are decomposed by data features and fused clustering algorithm to realize the cultural differences on the perspective of linguistic and cultural communities.

The article "Modeling and Analysis of the Influence of Cultural Differences on English Learning from the Perspective of the Cultural Community" was published in 2022. Journal: J Environ Public Health.

## 5. Simulation and Test

A total of 60 students in two grade experimental classes with 30 students in each class were selected as test subjects. The simulation experiment is carried out in the MATLAB environment with the computer operating system of Windows 10 and the memory of 4 G. In the experimental study, the personal characteristics of students are mainly the time data of students' landing on the platform. The learning time recorded by the “ability sky” platform mainly refers to the online time of students. By recording the login time of students on the platform, teachers can know whether the learning time of students meets the actual needs. According to the test and analysis of MATLAB platform, the data table of students' login time is derived, and the students are numbered in turn. The details of the learning time of 60 students on the platform are shown in Figure 4.

According to Figure 4, more than 95% of students are satisfied with the teaching resources and teaching environment arranged by teachers and are willing to use the “Ability Sky” platform to help them complete their courses. The “Ability Sky” platform can help them acquire, internalize, and consolidate their current knowledge; enhance their interest in English learning and learning efficiency with the help of the “Ability Sky” teaching platform; promote personalized learning; and help students learn a lot through teachers' analysis and feedback of personalized data. From the students' attitude towards the implementation of teaching, it can be seen that the junior high school English learning through the “Ability Sky” teaching platform is helpful to their individualized learning.

Students' personalized learning methods based on online teaching platform can analyze the contribution level of cultural differences to English learning, as shown in Figure 5.

It can be seen from Figure 5 the western culture. The Eastern culture or African culture, the personalized learning method of students using the online teaching platform, has a contribution weight of more than 75 to English learning up to 90. The contribution of this method to Oriental culture and African culture is particularly obvious, with an average value of about 85.

At different levels of differences, the accuracy of the evaluation of the influence of different cultural differences on English learning is tested, and the comparison results are shown in Figure 6.

It can be seen from the image comparison results in Figure 6 that the accuracy of the methods in this paper is above 90%, up to 100%, and the average value is about 95%. Compared with the two methods, the accuracy of the linear equalization algorithm is 70% ~90%, and the average accuracy is about 85%. The evaluation accuracy of analytical regression calculation is the lowest, ranging from 60% to 70%, and the average accuracy is 65%. By comparing the three methods, we can see that the accuracy of this method is the highest, which proves that the accuracy of this method is higher.

The article "Modeling and Analysis of the Influence of Cultural Differences on English Learning from the Perspective of the Cultural Community" was published in 2022. Journal: J Environ Public Health.

Based on the analysis of students' achievement, English learning attitude, and English learning strategies and questionnaires, it can be seen that the individualized learning of junior high school English supported by the network teaching platform has not greatly improved students' English achievement. However, through the comparison before and after the experiment, the individualized learning of junior high school English supported by the network teaching platform has greatly improved students' attitude towards English learning and learning strategies. Compared with before the experiment, students prefer learning English subjects. Through the questionnaire, it can be seen that the overwhelming majority of students like individualized learning of junior high school English supported by online teaching platform not only pays attention to their learning style but also effectively combines their interests with English learning. The personalized learning of junior high school English supported by the network platform enriches the traditional evaluation methods and objectively evaluates individual learning through personalized data. In addition, students can objectively understand their own learning situation through the learning process data recorded on the platform and the analysis results of the data and students can find their own shortcomings in learning and adjust their learning methods in time according to the feedback of personalized data.

## 6. Conclusions

This paper presents a model of the influence of cultural differences on English learning from the perspective of language and culture community based on data feature decomposition and fusion clustering. Relevant data are collected on the English learning platform, including learners' learning logs and learning achievements. From the perspective of language and cultural community, the quantitative analysis of the impact of cultural differences on English learning is realized. According to the analysis results of the simulation test, the personalized learning of junior high school English supported by the network teaching platform has greatly improved students' attitudes and learning strategies towards English learning. The model of the influence of cultural differences on English learning from the perspective of language and culture community established by this method has good data fusion performance, and the quantitative analysis results are accurate and reliable. It is hoped that in the future research, this method can be applied to the teaching of other subjects to cultivate excellent students with all-round development.

The article "Modeling and Analysis of the Influence of Cultural Differences on English Learning from the Perspective of the Cultural Community" was published in 2022. Journal: J Environ Public Health.

## Figures and Tables

**Figure 1:** The process of feature matching model construction.

**Figure 2:** The process of extracting feature information.

**Figure 3:** The process of decomposition of correlation characteristics.

**Figure 4:** Time chart of students' landing study.

**Figure 5:** The influence of difference contribution level.

**Figure 6:** Comparative test on the accuracy of evaluation.

## Data Availability

The raw data supporting the conclusions of this article will be made available by the authors, without undue reservation.
